RETRACTED

# Treatment of Upper Cervical Spinal Cord Injury (Unstable C1-C2) by Direct Visualization and Nailing Technique and the Advantages of Early MRI

**DOI:** 10.1155/2021/4562618

**Published:** 2021-09-29

**Authors:** Jamal Alshorman, Lian Zeng, Yulong Wang, Fengzhao Zhu, Kaifang Chen, Sheng Yao, Xirui Jing, Yanzhen Qu, Tingfang Sun, Xiaodong Guo

**Affiliations:** Department of Orthopedics Union Hospital Tongji Medical College, Huazhong University of Science and Technology, Wuhan 430022, China

## Abstract

**Background:**

The treatment of C1-C2 fractures mainly depends on fracture type and the stability of the atlantoaxial joint. Disruption of the C1-C2 combination is a big challenge, especially in avoiding vertebral artery, nerve, and vein sinus injury during the operation.

**Purpose:**

This study aims to show the benefit of using the posterior approach and pedicle screw insertion by nailing technique and direct visualization to treat unstable C1-C2 and, moreover, to determine the advantages of performing early MRI in patients with limited neck movement after trauma.

**Method:**

Between Jan 2017–Feb 2019, we present 21 trauma patients who suffered from C1, C2, or unstable atlantoaxial joint. X-ray, computed tomography (CT), and magnetic resonance image (MRI) were performed preoperatively. All the patients underwent our surgical procedure (posterior approach and pedicle screw placement by direct visualization and nailing technique).

**Result:**

The mean age was 41.1 years old, 8 females and 14 males. The average follow-up time was 2.6 years. Four patients were with C1 fracture, seven with C2 fracture, six with atlantoaxial dislocation, and four with C1 and C2 fractures. The time of MRI was between 12 hours and 48 hours; neck movement symptoms appeared between 2 days and 2 weeks.

**Conclusion:**

The posterior approach to treat the C1 and C2 fractures or dislocation by direct visualization and nailing technique can reduce the risk of the vertebral artery, vein sinus, and nerve root injuries with significant improvement. It can show a better angle view while inserting the pedicle screws. An early MRI (12–48 hours) is essential even if no symptoms appear at the time of admission, and if it is normal, it is necessary to repeat it. The presence of skull bleeding can be associated with upper neck instability.

## 1. Introduction

Many techniques were performed across the past years to treat atlantoaxial instability [1]. Posterior pedicle screw fixation has been a standard treatment of atlantoaxial instability [2–5]. However, the precise and safe placement of atlantoaxial pedicle screws in C1 and C2 remains challenging because of the complex anatomy [2]. C2 nerve root and vertebral artery injuries during pedicle screw placement have been stated in various studies [5]. The atlantoaxial fracture and instability can happen by multiple causes (trauma, degenerative disease, or malignancy) and commonly be stabilized by posterior fixation [6]. Resnick and Benzel first introduced screw placement in the atlas vertebra through the posterior arch and lateral mass [7]. Tan et al. first introduced the C1 pedicle screw fixation technique [8]. Biomechanical studies showed that C1 pedicle and lateral mass screws have greater stiffness [9]. At the same time, the method is often used for C1-C2 instability, and it demands fluoroscopic guidance, which needs a longer operation time and has high risks of radiation exposure [10]. Posterior pedicle screw placement has many advantages includeing better view, high fusion rate, fewer complications, less venous bleeding, more significant cortical purchase, and longer screw length than the atlas lateral mass screw procedure, which make it more suitable for short-segment fixation [4, 11, 12]. Simultaneously, considering a safe screw entry point on the C1 posterior arch, similar to the C2 posterior arch screw technique, can provide adequate biomechanical stability [13]. This study shows the effectiveness of direct visualization and nailing techniques in treating C1-C2 instability by safe entry points of pedicle screws and the importance of early MRI.

RETRACTED

### 1.1. Patients Characteristics and Method

Between January 2017 and February 2019, 21 trauma patients came to our department (Orthopedics Department of Union Hospital, Tongji Medical College) complaining of severe neck pain and neck movement limitation. Some were sent from another institute for further treatment; two patients came with neck support and immobilization. All the patients were with unstable C1-C2, which required surgical treatment. All patients underwent a posterior approach procedure and insertion pedicle screw by direct visualization and nailing technique. The posterior vertebral arch was less than 4 mm in all patients.

### 1.2. Statistical Analysis

SPSS statistical software (IBM version 22) was used to analyze the collected data: age, gender, mechanism of injury, fractured vertebrae, time of MRI, time of symptoms appearance, and the number of fusion vertebrae. Variables are presented as numbers and percentages. Unpaired *t*-test was used. The *P* value <0.05 was considered to be statistically significant.

### 1.3. Anatomy of C1-C2

Different vertebral arteries were classified at the craniovertebral junction, and the most common type was the high-riding vertebral artery. The injury of the C2 artery will be at high risk when the C2 height and width is less than 4mm and with high-riding vertebral artery type.[14]. Moreover, 3D preoperative planning can help understand the exact anatomy of C1 and C2 in each patient, reducing the risk of vertebral artery injury, as well as measuring the C2 isthmus height and width; understanding the detail of the morphological isthmus features can decrease the risk of vertebral artery injury and make the surgeon aware in some cases. C1 cover parts of the odontoid process [15], so it is essential to identify the exact problem in upper SCI and the presence of other abnormalities (bone fragments and degree of displacement). The complexity of C1 and C2 structure reveals that surgical procedure is a better choice that improves the stability of the C1-C2 combination.

RETRACTED

### 1.4. Preoperative Examination

After trauma, all the patients who came to our department underwent neck support and immobilization until the operation time. X-ray, CT, and MRI were performed preoperatively to check the patient's condition: atlantoaxial joint stability, cervical vertebral sequences, neck curvature, presence of edema or hemorrhage, soft tissue injury, and bone fragments in spinal canal. Heart rate, pulse, respiratory rate, temperature, and blood test were examined to check the patient's hemostasis and chest, back, upper, and lower extremities for other associated injuries. Motor and sensory functions of the upper and lower limbs and perianal reflux were checked. Hoffman's sign, bilateral knee-tendon reflex, Achilles tendon reflex, bilateral ankle clonus, and Babinski's sign were examined in all patients. Range of neck movement was used to assess the neck function.

### 1.5. Surgical Technique

The patient was located in the prone position after receiving general anesthesia, and the neck was slightly flexed for a better view, and the head holder was applied. A midline incision was done; the fascia and muscle were dissected to expose the C1 and C2 posterior arch.

The posterior arch (C1 and C2) was fully exposed using subperiosteal dissection. Two dissectors were inserted carefully along the surface of the C1 posterior arch; the vertebral artery was protected at the vertebral artery groove's surface, and the C2 vein and nerve root were carefully managed and pushed away from the inferior edge for a distance of approximately 3 mm. C1 nail placement is arranged to determine the pedicle's width and direction, and the inward and upwardly inclined needle insertion angles are determined.

The C1-C2 posterior arch was assessed for any deformity under direct vision and posterior arch height (posterior arch height was <4 mm in all patients) at the vertebral artery groove (Figure 1). The posterior arch was dissected with great attention and the first to look for dural venous plexus injured or not. The entry point at the C1 posterior arch was approximately 1.8–2 cm lateral to the midline. According to preoperative CT scans and intraoperative anatomy, the optimal direction of the trajectory was made. The surgical nail was used gently with sufficient, safe, and effective mechanical strength to penetrate the hard cortical bone and preventing the disc from moving backward and create another spinal cord injury. The direction of nail insertion was under direct vision, but, before inserting the screw, the direction was confirmed by fluoroscopy. A probe was used to approximately 4 mm at the posterior arch inferior to the vertebral artery groove along the path that can expose the feasible screw entry point (Figure 2). Bone graft was modified to implant on the posterior rim of C1 and C2. The neck circumference was externally fixed after the operation; the lateral position was preferred to avoid more pressure at the injury site.

RETRACTED

## 2. Result

Twenty-one patients underwent internal fixation by a posterior approach using internal screw fixation by direct visualization and nailing techniques after trauma. Eight females and thirteen males included in this study. The younger patient was 13 years old, and the older patient was 57 years old with a mean age of 41.1 years old. Seven patients were presented after fall from a height and 14 after road traffic accident. Twenty patients were treated through C1-C2 internal fixation, one with C1-C3 and one required laminectomy (Table 1). Ten patients had associated fractures (skull, ribs, scapula, femur, radius, and thoracic and lumbar vertebrae). After the operation, postoperative radiographic and CT scans confirmed that all pedicle screws were inserted successfully in all patients. After the procedure, motor and sensory functions improved in all the patients, and there was no complication and no artery or nerve injury. Also, all the patients showed good improvement, except one that remained paraplegic, but the feeling and movement improved slightly.

At last, a solid bone union was achieved in all patients, and there were no hardware failures. The time of MRI was between 12 hrs and 48 hrs, except in two patients who underwent MRI in other institutes. Neck symptoms appeared between 2 days and 2 weeks, but in one patient, it takes more than a month to complain of limited neck movement. All the patients' postoperative MRIs showed the disappearance of edema, hemorrhage, and spinal cord compression.

## 3. Discussion

The atlas and axis bones anatomy is complex, and various nearby organs (artery, venous plexus, and nerve) make a complex procedure. Distal to the atlas bone, the pedicle is connected between the vertebral body and arch. Pedicle heights of the atlas are different between various patients [16]. However, taking a good viewpoint before opening the cortical bone can ensure the insert of the screw in the safe zone. Edema starts appearing 12 hours after the onset but at the upper cervical spinal canal (C1-C2) is widest, so it may take a longer time to collect fluids (edema or hemorrhage) to increase the pressure around the cord (spinal cord compartment syndrome) which delays the symptoms appearance [17]. Moreover, this can increase the chance of secondary injury. The symptoms will be less severe and dangerous as space is more expansive at C1-C2, so performing early MRI (12–48 hours) and using DTI with DTT can show the severity of the injury and the collection of fluids and blood and classify the injury severity and show more pathological details. Moreno et al. presented a case report after trauma with atlantoaxial subluxation [18]. However, other pathological changes appeared after a long time. Stenosis at C1-C2 can cause venous hypertension and congestion and might lead to hemorrhage after a long time of the onset. Moreover, MRI revealed lesions with acute cervical myelopathy. Performing an early MRI and repeating it after normal appearance are very important. Using another technique such as diffusion tensor imaging (DTI) and diffusion tensor tractography (DTT) will have significant advantages in showing the micropathological changes in the spinal cord white matter. The exact time to perform MRI and other examination techniques can evaluate the pathological changes around the cord and choose the appropriate treatment, and starting early treatment will significantly improve the results.

RETRACTED

Cruciate and alar ligaments support the atlas bone, so disruption of the atlas's stability affects the axis to a large extent. Comminuted or unstable fractures treated by traditional methods or external immobilization can cause complications such as kyphosis, pseudarthrosis, and nonunion [19]. However, if the fracture is stable, then immobilization and cervical collar can be used, bearing in mind other abnormalities (disc herniation of a distal vertebra or bone fragment in the spinal canal) that are indications for surgery. For better and faster recovery and to avoid additional complications, then surgical procedure is a better choice. The fracture's stability dictates the management of unstable spine fracture that causes progressive pain, neurological deficit, spine deformity, fracture with hemorrhage or edema, or fracture with soft tissue injury descend under different managements [17]. The posterior pedicle screw placement technique may be an effective and reliable option for unstable atlas and axis fractures.

High force injury can cause edema or hemorrhage around the spinal cord. In this study, preoperative MRI showed edema in four patients and hematoma in two. In comparison, one patient had an extensive hematoma that required laminectomy. A hemorrhage or extensive edema is an urgent condition that needs to be evacuated to achieve a good prognosis and prevent more damage. However, MRI can be normal in few cases, so it is essential to understand the mechanism of the injury and patient's trauma history. Furthermore, using DTI and DTT to classify the injury severity can help determine the diagnosis and predict the prognosis [20, 21]. The preoperative management should be based on the patient's medical history, CT, and MRI.

The pathological changes on MRI correlated with the initial neurological defect [22]. However, in our study, the symptoms of unstable C1-C2 appeared between 2 days and 2 weeks, which means neck symptoms in some patients after trauma will not appear immediately. After trauma, the surgeon will focus on the upper or lower extremities, delaying the finding and treating the C1-C2. The presence of brain hemorrhage can be associated with disruption of the upper cervical fracture. So, performing MRI after high energy trauma significantly benefits in finding upper cervical pathological changes. MRI documentation of the spinal cord compression altered the time of surgical intervention. It can show the intra-axial hematoma, length of cord hematoma, progressive cord edema, spinal cord compression by extra-axial hematoma, and progressive neurological defect.

In severe injuries, the edema and hematoma can appear and increase in the first 48 hours and decrease gradually in the next three weeks, while hematoma indicates that Asia grade in the patient is A, or B, or some patients with C grade [23]. Grade A and B and neurodegenerative disorders at admission affect the prognosis [24]. Whatever is fractured type affected the C1-C2 stability. The main steps to achieve safe and stable screw placement are by measuring the height of the posterior arch and finding the safe screw entry point. Taking the transverse foramen as an accessory landmark can significantly benefit finding the entry point as the vertebral artery passes through it, putting the vertebral artery at higher risk of being injured. Using fluoroscopy for guidance is feasible and can show the safe direction of screws, especially in patients with posterior arch <4 mm. Complete or incomplete ponticulus posticus and a retrotransverse foramen or groove can be utilized as an accessory marker to clarify the entry point before screw placement [25]. In this study, a transverse foramen was taken as a landmark to protect the vertebral artery and refine the screw entry point by nail technique (Figure 3).

RETRACTED

Anterior and posterior approaches have few complications, but the posterior approach has some advantages over anterior, especially in stability. Treatment of unstable hangman's fracture is still controversial [26]. Posterior C1-C2 pedicle screw fixation can reduce complications, achieve high fusion rates, and expect excellent outcomes. In contrast, greater satisfaction for atlantoaxial fusion with a higher fusion rate than occipitocervical fusion limits cervical motion [27, 28]. The surgeons' concerns are to find the better treatment option to achieve faster and significant outcomes. Compression fracture of the atlas ring, or displacement of C1 more than 2 mm beyond the margin of C2, or tension band disruption must be treated by surgical intervention [29]. Further, the unstable odontoid fractures (type 2 and 3) must be treated by internal fixation technique to manage C1-C2 instability. Neurological deterioration at the time of onset is a landmark of spinal abnormalities [30–32]. The presence of associated fractures with neck pain (skull, ribs, scapula, femur, radius, thoracic vertebrae, and lumbar vertebrae) means high force energy trauma can be an accessory mark for unstable C1-C2, which require fast management. Six patients in this study did not show any symptoms at the onset. Some factors such as extensive edema, hematoma, and spinal stenosis compressed the vertebral artery, vein, and nerve and might cause venous hypertension and congestion and lead to venous damage and cause further complications. While looking forward to finding the screw entry point and protection, the vertebral artery is the main point to avoid intraoperative complications.

There are a few limitations of this study that we present in small sample size. Five patients came late to our department, three one week after injury, and one almost after a month and remained paraplegic with a slight improvement in motor and sensory functions after laminectomy and internal fixation.

## 4. Conclusion

Atlas or axis fractures, dislocation, fragment bone in the spinal canal, severe canal stenosis, compressed vertebral artery, disc herniation, hematoma, and extensive edema require surgical intervention. Our data and the internal fixation surgical nailing procedure make it feasible to treat the unstable C1-C2 fractures or dislocation without intraoperative complications. Using the nailing technique can easier determine the pedicle's width, direction, and insertion angle, indicate better intraoperative view at the screw entry point, and reduce the risk of other component injuries (vertebral artery, nerve, and venous sinus) even though posterior arch height <4 mm. Moreover, skull fracture or brain hemorrhage can be associated with C1-C2 instability in trauma patients; other fractures can mimic the C1-C2 instability and delay the diagnosis. Postoperative CT can ensure the stability of screws. Performing MRI in trauma patients in the first 12–48 hours can show the severity and the stability of C1-C2. Using DTI-DTT can ensure the injury severity and determine the diagnosis and predict the prognosis.

RETRACTED

## Figures and Tables

**Figure 1:** The posterior direct visualization approach combined with pedicle screw fixation by nailing technique. A patient with C1-C2 instability underwent posterior internal fixation and screw placement. (a) The incision site and dissecting the muscles; (b) a method of protecting vertebral artery, nerve, and venous sinus, before opening the screw entry point; (c) the screw entry point in the cortical bone after using a surgical nail; (d) postoperative after screw placement.

**Figure 2:** The nailing technique from left to right. As we reach the vertebral groove, the next step will protect the vertebral artery, venous plexus, and nerve root; we will finally open the cortical bone at the safe point and insert the screw. However, before inserting the screw, we confirm the direction under fluoroscopy.

**Figure 3:** The vertebral body where the posterior arch <4 mm. (a) The safe zone of inserting the screw; (b) the nail opening the cortical bone before inserting the screw.

**Table 1:** The patients' data included age, gender, fracture site, and treatment area. All the patients underwent posterior approach and pedicle screw placement by direct visualization and nailing technique.

Age	Gender	Fracture level	Treatment type
51	M	C2	C1 + C2
56	F	C2	C1 + C2
29	F	C1	C1 + C2
59	M	Atlantoaxial dislocation	C1 + C2
52	M	C2	C1 + C2
13	F	Atlantoaxial dislocation and odontoid fracture type 3	C1 + C2
49	F	C1	C1 + C2
29	F	Atlantoaxial dislocation	C1 + C2
54	M	C1 + C2	C1-C3
33	M	C1	C1 + C2
48	M	C1 + C2 fracture and subluxation	C1 + C2
39	M	Odontoid fracture type 3	C1 + C2
52	M	C1 + C2 and atlantoaxial subluxation	C1 + C2
31	F	Odontoid fracture type 3 and atlantoaxial dislocation	Laminectomy and hematoma removal at C1-C4
24	F	C1 + C2	C1 + C2
36	M	C2	C1 + C2
50	M	C2	C1 + C2
25	F	Atlantoaxial dislocation	C1 + C2
33	M	C1	C1 + C2
54	M	Base odontoid fracture	C1 + C2
57	M	Base odontoid fracture and right transverse foramen	C1 + C2

M, male; F, female.

## Data Availability

The study cases were collected from the Orthopedics Department at Union Hospital of Tongji Medical College.
